This article has been retracted.

# Increased Age-Adjusted Cancer Mortality After the Third mRNA-Lipid Nanoparticle Vaccine Dose During the COVID-19 Pandemic in Japan

**DOI:** 10.7759/cureus.57860

**Published:** 2024-04-08

**Authors:** Miki Gibo, Seiji Kojima, Akinori Fujisawa, Takayuki Kikuchi, Masanori Fukushima

**Affiliations:** 1 Primary Health Care, Matsubara Clinic, Kochi, JPN; 2 Pediatrics, Nagoya Pediatric Cancer Fund, Nagoya, JPN; 3 Cardiovascular Medicine, Honbetsu Cardiovascular Medicine Clinic, Honbetsu, JPN; 4 Translational Research & Health Data Science, Learning Health Society Institute, Nagoya, JPN

**Keywords:** breast cancer, prostatic carcinoma, pancreas tumors, oral cancers, leukemia, ovarian cancers, excess mortality, covid-19, sars-cov-2 mrna vaccine, age-adjusted mortality rate

## Abstract

During the COVID-19 pandemic, excess deaths including cancer have become a concern in Japan, which has a rapidly aging population. Thus, this study aimed to evaluate how age-adjusted mortality rates (AMRs) for different types of cancer in Japan changed during the COVID-19 pandemic (2020-2022). Official statistics from Japan were used to compare observed annual and monthly AMRs with predicted rates based on pre-pandemic (2010-2019) figures using logistic regression analysis. No significant excess mortality was observed during the first year of the pandemic (2020). However, some excess cancer mortalities were observed in 2021 after mass vaccination with the first and second vaccine doses, and significant excess mortalities were observed for all cancers and some specific types of cancer (including ovarian cancer, leukemia, prostate cancer, lip/oral/pharyngeal cancer, pancreatic cancer, and breast cancer) after mass vaccination with the third dose in 2022. AMRs for the four cancers with the most deaths (lung, colorectal, stomach, and liver) showed a decreasing trend until the first year of the pandemic in 2020, but the rate of decrease slowed in 2021 and 2022. This study discusses possible explanations for these increases in age-adjusted cancer mortality rates.

## Introduction

The COVID-19 pandemic began in December 2019 in Wuhan, China, and was first detected in Japan in January 2020. In response, a range of healthcare and socio-economic restrictions were implemented to curb the spread of the disease. Since February 2021, the mRNA-lipid nanoparticle (mRNA-LNP) vaccine has been available for emergency use and is recommended for all individuals aged six months and older, especially those at high risk. As of March 2023, 80% of the Japanese population had received their first and second doses, 68% had received their third dose, and 45% had received their fourth dose [1]. Despite these national measures, 33.8 million people had been infected, and 74,500 deaths had been attributed to COVID-19 in Japan by the end of April 2023. Additionally, excess deaths from causes other than COVID-19 have been reported in various countries [2-6], including deaths from cancer [7-10], and Japan is no exception [11,12]. Cancer is the leading cause of death in Japan, accounting for one-fourth of all deaths. Therefore, it is essential to understand the effects of the pandemic on mortality rates of cancer from 2020 to 2022. Age adjustment is necessary for accurate evaluation, especially in diseases such as cancer that tend to occur in elderly adults. Japan has several characteristics that make it ideal for analyzing the impact of the pandemic on cancer mortality rates, including its large population of 123 million, availability of official statistics, and the high 80% accuracy rate of death certificates according to autopsy studies [13].

## Materials and methods

Statistical data

The data used in this analysis are all publicly available national data. Death figures were obtained from the Vital Statistics [14], which include monthly and annual deaths by cause, sex, and age (five-year age groups). Cancer deaths are divided into 20 subclassifications. Only Japanese individuals living in Japan are included. Population estimates by age group required for the age-adjusted analysis were also obtained from the national data [15]. The number of people with confirmed COVID-19 infection was obtained from the Ministry of Health, Labour and Welfare website [16]. Vaccination rates by age group were obtained from the websites of the Prime Minister's Office and the Ministry of Health, Labor and Welfare [1,17].

Age-specific mortality rate (ASMR)

Annual crude numbers of deaths were grouped by 10-year age groups for the 0-39 age range, which had fewer deaths, and in five-year age groups for the 40-89 age range, which had more deaths. However, due to the small sample size, ages 90 and older were combined into one group.

ASMR (per 100,000 people)$\small = d_{}i\div p_{i}\times 100,000$

d_i_=crude number of deaths in that age group, p_i_=number in that age group in the observed population

Age adjustment by direct standardization

Because ASMRs are too detailed to provide an overview of mortality for all cancers, we used the age-adjusted mortality rate (AMR) from direct standardization as a summarized indicator. For comparisons of mortality rates over time, as in our study, all data are from the Japanese population as a whole, with comparably large numbers and age composition. The specific death rates per age group are known, so direct standardization is appropriate [18]. The Ministry of Health, Labour and Welfare in Japan reportedly uses direct standardization with smoothed standard population data from 2015 (125.32 million) [19], and the same approach was used in this study. The formulas for the calculation are as follows:

age-adjusted number of deaths $\small =\sum \left ( d_{i}\div p_{i}\times ps_{i} \right )$

age-adjusted mortality rate(AMR) (per 100,000 people）$\small =\sum \left ( d_{i}\div p_{i}\times ps_{i} \right )\div \sum ps_{i}\times 100,000$

i=age group, d_i_=number of deaths in that age group, p_i_=number in that age group in the observed population, ps_i_=number in that age group in the standard population.　　

Age adjustment for sex-specific cancers was performed using the “sex-specific smoothed standard population dataset 1” [20]. In leap years, the deaths had occurred in 366 days, so the age-adjusted number of annual deaths and AMR were multiplied by 365/366 to correct. The age-adjusted number and rate of deaths in February in leap years were also corrected for monthly analysis.

Excess mortality during the COVID-19 pandemic

Excess mortality in this study was defined as follows:

Excess number of deaths$= Do\, -\, Dp$

D*o*=observed number of deaths, D*p*=predicted number of deaths in the corresponding year or month 

Excess mortality (%)$= \left ( Ro\, -\, Rp\right )\div Rp\times 100$

R*o*=observed rate, R*p*=predicted rate in the corresponding year or month (rate is ASMR or AMR)

The predicted rates based on the 2010-2019 period before the COVID-19 pandemic were calculated using logistic regression analysis [5]. The predicted AMRs for each month were also calculated using data from the corresponding month in 2010-2019. R (version 4.3.1; R Development Core Team, Vienna, Austria) was used for statistical analysis.

The confidence intervals (CIs) and prediction intervals (PIs) around the predicted rates were calculated by logit-transformed values using the following formulas and then transformed inversely.

residual variance (σ^2^)$\small =\sum \left ( Vo_{i}\, -\, Vp_{i}\right)^{2}\div \left ( n-p-1 \right )$

standard error (SE_i_) for logit-transformed confidence interval (l-CI)$\small =\sqrt{\sigma ^{2}\times\left ( \frac{1}{n}+\left ( x_{i}-\bar{x} ^{}\right ) ^{2}\div \sum\left ( x_{i}-\bar{x} \right )^{2} \right )}$

standard error (SE_i_) for logit-transformed prediction interval (l-PI)$\small =\sqrt{\sigma ^{2}\times\left (1+ \frac{1}{n}+\left ( x_{i}-\bar{x} ^{}\right ) ^{2}\div \sum\left ( x_{i}-\bar{x} \right )^{2} \right )}$

logit-transformed CI (l-CI) or PI (l-PI) = Vp_i_ ± t_n-p-1_(probability)$\small \times SE_{i}$

Vo_i_ =logit-transformed ASMR or AMR, Vp_i_=logit-transformed predicted ASMR or AMR, n =number of observations (here, it is 10; from 2010 to 2019), p =number of explanatory variables (here, it is 1), x_ i_ =current year (here, it is one of 2010,2011,･･･,2022), $\small \small \bar{x}= \sum x_{i}\div n$, t_n-p-1_ (probability) =t value at the degree of freedom (n-p-1), and the probability of interest

## Results

Mortality from all causes and all cancers

Table 1 shows the numbers of crude, age-adjusted, and excess deaths for all causes, all cancers, and each cancer type with the excess mortality rates during the pandemic in 2020, 2021, and 2022. Each cancer type is listed in decreasing order of number of deaths in 2022. The annual numbers of age-adjusted deaths in 2020, 2021, and 2022 during the pandemic were 1,206,126, 1,244,976, and 1,320,768 from all causes, and 345,248, 345,625, and 344,114 from all cancers, respectively. In 2020, the first year of the pandemic, there was significant deficit mortality for all causes (< 99% lower PI) and no excess mortality for all cancers. However, in 2021, there was significant excess mortality of 2.1% (>99% upper PI) for all causes and 1.1% (>95% upper PI) for all cancers. In 2022, the excesses increased to 9.6% (>99% upper PI) for all causes and 2.1% (>99% upper PI) for all cancers. In 2022, the number of excess deaths was 115,799 (95%CI: 106,018, 125,501) for all causes and 7,162 (95%CI: 4,786, 9,522) for all cancers. Among the 20 subclassifications, the five cancers with the most deaths (lung, colorectal, stomach, pancreatic, and liver cancer) accounted for 61% of deaths from all cancers. The ranking of the number of deaths for each cancer type was nearly unchanged from 2020 to 2022.

**Table 1:** Observed crude, age-adjusted, and excess deaths for all causes, all cancers, and each cancer type with excess mortality rates during the pandemic in 2020, 2021, and 2022. Each cancer type is listed in decreasing order of the number of deaths in 2022. Excess mortality = (observed AMR - predicted AMR) / predicted AMR * 100 (%). (Predicted AMRs based on the pre-pandemic years 2010-2019 were calculated using logistic regression.) Symbol ⁑ for >99%, * >95% upper, ‡<99%, †<95% lower prediction interval (PI)

Cause of death and ICD-10 codes		Crude number of deaths			Age-adjusted number of deaths			Excess number of deaths (age-adjusted)			Excess mortality (age-adjusted)		
														2020	2021	2022	2020	2021	2022	2020	2021	2022	2020	2021	2022
		All-cause of deaths		1,372,648	1,439,809	1,568,961	1,206,126	1,244,976	1,320,768	-28,126	25,453	115,799	-2.3%‡	2.1%⁑	9.6%⁑
Malignant neoplasms C00-C97		378,356	381,497	385,787	345,248	345,625	344,114	-1,379	3,870	7,162	-0.4%	1.1%*	2.1%⁑
Subclassification	Malignant neoplasm of trachea, bronchus and lung C33–C34	75,581	76,212	76,664	68,721	68,832	68,292	-352	672	1,033	-0.5%	1.0%	1.5%
	Malignant neoplasm of colon, sigmoid, and rectum C18-C20	51,784	52,416	53,088	47,303	47,498	47,338	-859	-380	-259	-1.8%	-0.8%	-0.5%
	Malignant neoplasm of stomach C16	42,318	41,624	40,711	38,388	37,458	35,940	-199	366	286	-0.5%	1.0%	0.8%
	Malignant neoplasm of pancreas C25	37,674	38,578	39,468	34,590	35,249	35,593	296	651	688	0.9%*	1.9%⁑	2.0%⁑
	Other remaining malignant neoplasm in C00–C97	28,592	28,934	29,646	26,024	26,065	26,273	-115	149	579	-0.4%	0.6%	2.3%
	Malignant neoplasm of liver and intrahepatic bile ducts C22	24,839	24,102	23,621	22,561	21,708	20,960	-42	161	421	-0.2%	0.7%	2.0%
	Malignant neoplasm of gallbladder and other parts of biliary tract C23–C24	17,772	18,172	17,758	15,810	15,990	15,303	-255	333	43	-1.6%	2.1%	0.3%
	Malignant neoplasm of breast C50	14,650	14,803	15,911	14,089	14,185	15,109	-558	-631	122	-3.8%†	-4.3%†	0.8%
	Malignant lymphoma C81–C86	13,995	13,997	14,230	12,591	12,507	12,437	239	64	-98	1.9%	0.5%	-0.8%
	Malignant neoplasm of prostate C61	12,758	13,216	13,440	10,775	10,981	10,835	131	547	604	1.2%	5.3%*	5.9%*
	Malignant neoplasm of esophagus C15	10,978	10,958	10,918	10,298	10,248	10,105	-381	-226	-170	-3.6%	-2.2%	-1.7%
	Leukemia C91–C95	8,983	9,120	9,758	8,280	8,397	8,868	-16	143	656	-0.2%	1.7%	8.0%*
	Malignant neoplasm of bladder C67	9,166	9,443	9,597	8,060	8,196	8,114	-181	-68	-171	-2.2%	-0.8%	-2.1%
	Malignant neoplasm of lip, oral cavity and pharynx C00–C14	7,826	8,000	8,429	7,257	7,364	7,636	-46	92	395	-0.6%	1.3%	5.5%*
	Malignant neoplasm of uterus C53–C55	6,806	6,818	7,156	6,568	6,589	6,877	-73	-86	168	-1.1%	-1.3%	2.5%
	Malignant neoplasm of ovary C56	4,875	5,081	5,182	4,732	4,928	4,989	114	347	442	2.5%	7.6%⁑	9.7%⁑
	Other malignant neoplasms of lymphoid, hematopoietic,etc. C88–C90, C96	4,295	4,351	4,391	3,857	3,888	3,850	-136	-45	-22	-3.4%	-1.1%	-0.6%
	Malignant neoplasm of central nervous system C70–C72, C75.1–C75.3	2,847	3,054	3,106	2,729	2,944	2,966	-165	-46	-120	-5.7%	-1.5%	-3.9%
	Malignancy of skin C43–C44	1,707	1,718	1,806	1,532	1,512	1,546	8	1	47	0.6%	0.1%	3.2%
	Malignant neoplasm of larynx C32	781	795	798	714	721	707	-62	-27	-15	-8.0%	-3.6%	-2.1%

Figure 1 shows the annual AMRs over time and the excess mortality rates in each month during the COVID-19 pandemic (2020-2022) of all cancers. AMRs had been decreasing until 2020 (AMR 275.5/100,000 population), but this decline stopped after 2021, exceeding the 95% upper PI in 2021 (AMR 275.8/100,000) and the 99% upper PI in 2022 (AMR 274.6/100,000). As shown on the right side, the monthly excess mortality (%) exceeded the 99% upper PI for the first time in August 2021, coinciding with the peak of the first and second mass vaccinations and became elevated again from May 2022, two months later the peak of the third mass vaccination, once again exceeding the 99% upper PIs for four months until December.

**Figure 1:** Age-adjusted mortality rates (AMRs) over time and excess mortality in each month: all cancers. (Left side) Observed age-adjusted mortality rates (AMRs) (per 100,000 population) are represented by a blue line with marks, the predicted trend by logistic regression analysis by a dashed line, and the 95% prediction intervals (PIs) by dotted lines. Markers are highlighted in yellow for years with figures exceeding 95% of the upper PI, and pink for years with figures exceeding 99% of the upper PI. The vertical line indicates the arrival of COVID-19 in Japan. There was a decreasing trend until 2020, but the decline stopped after 2021, with figures exceeding the 95% upper PI in 2021 and the 99% upper PI (the line was not shown) in 2022. (Right side) The horizontal axis indicates each month during the pandemic in 2020, 2021, and 2022, while the vertical axis on the left side indicates the excess mortality (%), calculated as (observed AMR − predicted AMR in the corresponding month) / predicted AMR in the corresponding month*100. The predicted AMRs based on the 2010–2019 period preceding the COVID-19 pandemic were estimated by logistic regression analysis. The ⁑ symbol signifies >99% upper PI, and † <95% lower PI. The vertical axis on the right side indicates the number of domestic vaccinations and deaths attributed to COVID-19. Monthly excess mortalities exceeded the 99% upper PI for the first time in August 2021, coinciding with the peak of the first and second mass vaccinations, and once again exceeded the 99% upper PI for four months from May 2022, two months after the peak of the third mass vaccination.

Age-specific mortality for all cancers

Prior to the pandemic (2010-2019), crude age-specific mortality rates for all types of cancer had decreasing trends in all age groups, except for the 90+ age group (data not shown). In 2020, deficit mortality was observed in most age groups, except the 75-79 age group. However, this gradually shifted to excess mortality in 2021 and escalated in 2022 in almost all age groups, except for the 65-69 and 85+ groups. In the 75-79 age group, excess mortality was 3.9% (95%CI: 2.6, 5.3) in 2020, 7.9% (6.4, 9.5) in 2021, and 9.5% (7.8, 11.4) in 2022, each exceeding the 99% upper PIs. In the 80-84 age group, excess mortality was 2.9% (1.4, 4.5) in 2022, exceeding the 95% upper PI. No statistical significance was detected in the younger age groups, which had few deaths. The chart below shows that the number of deaths from all cancers was highest in the 80-84 age group (Figure 2). According to Table 2, more than 90% of people aged 70 and older have received a third vaccine dose [1,17]. The Ministry of Health, Labour and Welfare reported that more than 99.9% of formulations administered were mRNA-LNPs, with BNT162b2 accounting for 78.1% and mRNA-1273 accounting for 21.8% [17], up to third doses with monovalent vaccine.

**Figure 2:** Excess mortality during the pandemic in 2020, 2021, and 2022 (upper) and crude cancer deaths in 2022 (lower) in each age group. Excess age-specific mortality = (observed ASMR − predicted ASMR) / predicted ASMR * 100 (%). Predicted ASMRs based on the 2010-2019 period preceding the COVID-19 pandemic were calculated using logistic regression. The ⁑ symbol signifies >99% upper PI, * >95% upper PI, and †<95% lower PI. 2020, deficit mortality was observed in most age groups except for the 75–79 age group. However, mortality increased gradually in 2021 and more remarkably in 2022 in almost all age groups except for the 65–69 and 85+ age groups. In the 75–79 age group, excess mortality was 3.9% (95%CI: 2.6, 5.3) in 2020, 7.9% (95%CI: 6.4, 9.5) in 2021, and 9.5% (95%CI: 7.8, 11.4) in 2022, exceeding the 99% upper PIs. In the 80–84 age group, excess mortality was 2.9% (1.4, 4.5) in 2022, exceeding the 95% upper PI. No statistical significance was detected in the younger age groups, which had few deaths. The chart below shows that the number of deaths from all cancers was highest in the 80–84 age group.

**Table 2:** Vaccination rate by age group as of March 2023. More than 90% of people aged 70 and older have received a third vaccine dose.

Age group (year old)	6 month-4^※^	5-11	12-19	20-29	30-39	40-49	50-59	60-69	70-79	80-89	90-
First and second doses	3.1%	16.2%	67.4%	80.2%	80.5%	82.9%	90.7%	91.5%	93.7%	97.7%	99.3%
Third dose	0.9%	8.1%	42.8%	56.1%	58.8%	65.0%	79.0%	86.5%	91.1%	95.1%	96.0%

Mortality by cancer type

Figure 3 illustrates excess mortality for each type of cancer. In 2020, only pancreatic cancer slightly exceeded the 95% upper PI. However, statistically significant excess mortality was observed for three out of 20 types of cancers in 2021, and five out of 20 in 2022. The types were ovarian cancer, leukemia, prostate cancer, lip/oral/pharyngeal cancer, and pancreatic cancer, in descending order in 2022. AMRs exceeded the predicted value by 7.6% (95%CI: 5.6, 9.5) in 2021 and 9.7% (7.5, 12.0) in 2022 for ovarian cancer, 1.7% (-2.1, 5.7) and 8.0% (3.4, 12.8) for leukemia, 5.3% (2.7, 7.9), 5.9% (3.0, 8.9) for prostate cancer, 1.3% (-1.4, 4.1) and 5.5% (2.3, 8.7) for lip/oral/pharyngeal cancer, and 1.9% (0.4, 3.4) and 2.0% (0.3, 3.7) for pancreatic cancer. Breast cancer had significant deficit mortality in 2020 and 2021, which shifted to excess in 2022, though without statistical significance.

**Figure 3:** Excess mortality for each cancer type during the pandemic in 2020, 2021, and 2022. Excess mortality = (observed AMR − predicted AMR) / predicted AMR * 100 (%). Predicted AMRs based on the 2010–2019 period preceding the pandemic were calculated using logistic regression. The ⁑ symbol signifies >99% upper PI, * >95% upper PI, and †<95% lower PI. As shown on the far left, excess mortality from all cancers was observed in 2021 and 2022, each over the 95% or 99% upper PI. Of the 20 types of cancers, five showed significant excess mortality: these were ovarian cancer, leukemia, prostate, lip/oral/pharyngeal, and pancreatic cancers, in decreasing order of 2022 figures. Breast cancer had significant deficit mortality in 2020 and 2021, which then shifted to excess mortality, though without statistical significance.

AMRs for the four cancers with the most deaths (lung, colorectal, stomach, and liver cancer) showed decreasing trends until the first year of the pandemic in 2020, but the rate of decrease slowed in 2021 and 2022. Still, AMR stayed within the 95% PIs (Figure 4).

**Figure 4:** Trends in age-adjusted mortality rates over time for leading cancers (lung, colorectal, stomach, and liver). Lung, colorectal, stomach, and liver cancers all showed similar decreasing trends in age-adjusted mortality rates (AMRs). However, this decline slowed, and AMRs gradually exceeded the predicted values in 2021 and 2022 for all, except for colorectal cancer. Pancreatic cancer, the fourth leading cause of death, is described later.

Trends for cancer types with excess mortalities in 2021 and 2022

Five types of cancer, namely, ovarian cancer, leukemia, prostate, lip/oral/pharyngeal, and pancreatic cancer, had AMRs exceeding the predicted values in 2021 and/or 2022. Figure 5 illustrates the trends by year and month for these types of cancer. Four of them showed a gradual downward trend, while pancreatic cancer showed an upward trend over time. All five types of cancer showed an increase in 2021 compared to 2020, with ovarian, prostate, and pancreatic cancers exceeding 95% upper PIs in 2021, and all five cancer types exceeding 95% upper PIs in 2022. Monthly excess mortalities gradually rose for these cancers in 2021-2022 compared to 2020.

**Figure 5:** Age-adjusted mortality rates (AMRs) over time and excess mortality in each month for cancers with excess mortalities in 2021 and 2022. See Figure 1 for an explanation of the graphs' axes, units, and other elements. (A) Ovarian cancer There was a gradual downward trend from 2010, a slight increase from 2020, and a substantial increase from 2021 to 2022, with AMRs exceeding the 99% upper PIs in 2021 and 2022. Monthly excess mortalities gradually increased through 2021 and 2022. (B) Leukemia Annual AMRs of leukemia slowly declined or plateaued starting in 2010, but significantly increased in 2022, exceeding the 95% upper PI. Monthly AMRs exceeded the 99% upper PI in January and the 95% upper PI in December 2022. (C) Prostate cancer Annual AMRs were on a gradual downward trend starting in 2010, but increased starting in 2021, exceeding the 95% upper PIs in 2021 and 2022. Monthly excess mortalities gradually increased through 2021 and 2022, exceeding the 95% upper PI in December 2022. (D) Lip/oral/pharyngeal cancer Annual AMRs over time were on a gradual downward trend, but increased in 2022, exceeding the 95% upper PI. Monthly excess mortalities increased more clearly after the third mass vaccination for COVID-19 in 2022, exceeding the 95% upper PIs in January and December 2022. (E) Pancreatic cancer AMRs in 2015 were excluded from the analysis because it was an apparent outlier for unknown reasons. Annual AMRs of pancreatic cancer increased from 2010, began to exceed the 95% upper PI in 2020, and then deviated further and increased between 2021 and 2022, exceeding the 99% upper PIs. Monthly excess mortalities were seen from 2020, exceeding the 95% upper PI in December 2020, and increased even further, exceeding the 99% upper PIs in December 2021 and 2022.

Cancer type with monthly excess mortalities: breast cancer

Of the remaining 15 cancer types for which annual AMRs did not exceed the 95% PIs, the only cancer type for which monthly AMRs deviated from the 95% PIs multiple times in a year was breast cancer in women. Annual AMRs for breast cancer in women were under the 95% lower PIs in 2020 and 2021, and they increased in 2022 but remained within the 95% PI (Figure 6, left side). Monthly statistically significant excess mortality appeared several months after the peak of the third mass vaccination, exceeding the 95% upper PIs twice in 2022 (right side).

**Figure 6:** Age-adjusted mortality rates (AMRs) over time and excess mortality in each month during the pandemic: breast cancer. See Figure 1 for an explanation of the graphs’ axes, units, and other elements. Annual AMRs for breast cancer in women were under the 95% lower PIs in 2020 and 2021, and increased in 2022, but without statistical significance (left side). Monthly excess mortalities appeared several months later, after the third mass vaccination, exceeding the 95% upper PIs twice in 2022 (right side).

## Discussion

Scherb et al. estimated the crude excess mortality for all causes during the COVID-19 pandemic in Japan in 2020, 2021, and 2022 to be -2.84% (95%CI: -4.46, -1.25), 0.80% (-0.83, 2.40), and 8.37% (6.74, 9.97), respectively, using linear logistic trend predictions based on 2005 to 2019 [5]. In our study, we estimated age-adjusted excess mortality by logistic regression with predictions from 2010 to 2019 and calculated -2.3% (-2.7, -1.9), 2.1% (1.6, 2.6), and 9.6% (9.0, 10.2), respectively. These results seem consistent. For all cancers, we estimated the excess mortalities to be -0.4% (-0.9, 0.1), 1.1% (0.5, 1.8), and 2.1% (1.4, 2.8), respectively, indicating no excess in 2020 and statistically significant increases in 2021 and especially in 2022. 

Findings in 2020, during the first year of the pandemic

Mortality from all cancers did not increase in 2020. The only statistically significant deviations from the predictions in 2020 were a 3.9% excess in all cancer deaths among the 75-79 age group, a very slight (0.9%) excess in pancreatic cancer deaths, and a 3.8% deficit in breast cancer deaths (a 4.3% deficit in breast cancer deaths was also observed in 2021). In 2020, highly virulent strains of SARS-CoV-2 entered Japan, but there were relatively few deaths attributed to COVID-19 in Japan [21]. Declarations of pandemic emergency were issued three times before September 2021, requesting social distancing and securing hospitalization for COVID-19 patients. Modeling studies were conducted in some countries to estimate the impact of the pandemic on cancer mortality [7,8]. In fact, during the first wave of COVID-19 in Belgium in March and April 2020, cancer deaths increased by 10% and 33%, respectively, compared to the number of deaths predicted from 2013 to 2018 [9]. In Madurai, a south Indian city, deaths attributed to cancer increased 109% during the first weeks of lockdown [10]. In Brazil, during the first wave in March through May 2020, the numbers of biopsies, colonoscopies, mammograms, and oncological surgeries decreased by 29%, 57%, 55%, and 9%, respectively, compared to pre-pandemic figures. As a result, the number of hospitalizations for cancer decreased by 21%, whereas the mortality rate of hospitalized patients with cancer increased by 14% [22]. In Japan, the number of screenings for gastric, lung, colorectal, breast, and uterine cancers in the community decreased by 24.4% (at work, only 0.9%) in 2020 and appeared to have returned to original trends in 2021 [23]. The number of significant surgeries for gastrointestinal cancers decreased by 6.2% in 2020 and 5.1% in 2021 compared to those in 2018 and 2019 [23]. The decline of such cancer care could explain the excess cancer mortality among the 75-79 age group and the slight increase in pancreatic cancer deaths observed in 2020 in our study. The reasons for the decrease in breast cancer deaths in 2020-2021 are unknown.

Findings in 2021 and 2022, the second and third years of the pandemic 

The statistical findings on cancer deaths in 2021-2022 can be summarized as follows.

All cancer deaths: A statistically significant excess emerged in 2021 and increased further in 2022. In addition, significant excess monthly mortality was observed after August 2021, whereas mass vaccination of the general population began around April 2021. There were excess trends in cancer deaths across most age groups. However, these trends were only statistically significant for age groups with the highest cancer mortality: the 75-79 age group in 2021 and the 75-84 age group in 2022. More than 90% of people over 70 years of age have received the third vaccine dose.

Cancer type: Deaths from the most common types of cancer (lung, colorectal, stomach, and liver cancer) showed downward trends in the pre-pandemic period, and the rates of decrease slowed during the pandemic but remained within the 95% PIs. On the other hand, six of the 20 types of cancer (ovarian cancer, leukemia, prostate, lip/oral/pharyngeal, pancreatic, and breast cancer) had statistically significant excess mortalities in 2021, which increased further in 2022. Reduced cancer screening and healthcare due to the lockdown might increase deaths for any type of cancer. Still, the significant increases in mortalities for six specific cancer types were unlikely to be explained by a shortage of healthcare services. As for the incidences during this period, the crude numbers of all patients registered at core cancer care centers showed increasing trends for prostate cancer in men and breast cancer in women in 2021, especially in 2022 [24]. However, these are not age-adjusted and cannot be judged as increases.

Influence of multiple mRNA-LNP vaccine doses

Based on a report on domestic cancer care [23] and the absence of an emergency declaration from October 2021 onwards, the restrictions on access to cancer screening or treatment seem to have been much relieved after late 2021. Mass vaccination with the first and second doses started in the spring of 2021, and the vaccination rate soon peaked in the summer of 2021 at 80% of the population. The vaccination rate for the third dose peaked in the spring of 2022, at 68%. Now, Japan is even conducting mass vaccination with a seventh dose, making it the country with the highest vaccination rates.

Researchers have reported that the SARS-CoV-2 mRNA-LNP vaccine may pose the risk of development and progression of cancer [25-28]. In addition, several case reports have described cancer developing or worsening after vaccination and discussed possible causal links between cancer and mRNA-LNP vaccination [29-34].

Based on the molecular weight of BNT162b2 mRNA (Pfizer-BioNTech), the mRNA content per dose is estimated at 13 trillion molecules and 40 trillion molecules in mRNA-1273 (Moderna) [35,36]. The total number of cells in humans is estimated to be 37.2 trillion [37], making the number of mRNA-LNPs very high, ranging from one-third to the equivalent of the total cell number. After inoculation, the mRNA-LNPs are delivered to various organs, especially the liver, spleen, adrenal gland, ovary, and bone marrow [38]. In one study, vaccine mRNA was detected in the lymph nodes of persons vaccinated with hybridization of a SARS-CoV-2 mRNA vaccine-specific probe 7 to 60 days after the second mRNA-1273 or BNT162b2 dose [39]. Modified mRNA with N1-methyl-pseudouridine could translate a large amount of SARS-CoV-2 spike protein (S-protein) [40]. S-protein emerged on the surface of exosomes in the blood of the vaccinated [41]. Fragments of vaccine-specific recombinant S-protein were found in blood specimens of 50% of vaccine recipients and were still detected three to six months later [42].

On the other hand, in the case of SARS-CoV-2 infection, which is basically a respiratory infection, viral S-protein was only detected in serum for up to 10-20 days, even in patients with acute severe disease [43-45]. The attenuated Omicron strains emerged in Japan in early 2022 and have been prevalent at various points since then. As shown in the graphs in Figures 1, 5, and 6, the monthly number of vaccinated individuals was many times greater than that of newly confirmed cases of infection, and the cumulative number of vaccinated individuals (380 million) was 13 times that of newly confirmed cases of infection (30 million) until the end of 2022.

A study of more than 50,000 employees at a medical institution in the United States observed the incidence of the Omicron variant epidemic based on the number of vaccine doses received (0, 1, 2, 3, and 4 or more doses) over a period of 26 weeks and showed that the number of vaccines received was positively correlated with the cumulative incidence rate of COVID-19 [46]. Susceptibility to COVID-19 infection after multiple vaccinations may be enhanced by antibody-dependent enhancement [47], immune imprinting [39,48], and immunosuppression [25-27]. This can result in a risk of exposure to viral S-protein in addition to vaccine S-protein for the multiple-vaccinated. These data suggest a significant impact on vaccine recipients, including the large number of mRNA-LNPs that are injected, their rapid and widespread distribution particularly into specific organs, the amount of S-protein produced, its long persistence in the body, and increased susceptibility to infection. Next, we consider each factor that may contribute to the involvement of the mRNA-LNP SARS-CoV-2 vaccine in increasing mortality from all cancers and some specific cancer types.

Thrombogenic effects of spike protein and LNP

Because cancer often leads to the activation of coagulation via various mechanisms, one of the major causes of mortality in patients with cancer is cancer-associated thrombosis (CAT) [49-51], manifesting as disseminated intravascular coagulation (DIC) in its most extreme form [52]. Therefore, it is reasonable to assume that the additional thrombus-forming tendency noted with the mRNA-LNP vaccine could be extremely dangerous. The viral and vaccine S-protein of SARS-CoV-2, especially Omicron lineages, having a solid electro-positive potential, could attach to electro-negative glycoconjugates on the surfaces of red blood cells (RBCs), other blood cells, and endothelial cells [53]. The S-protein of SARS-CoV-2 alone has been reported to bind to angiotensin-converting enzyme 2 (ACE2) and activate angiotensin II receptor type 1 (AT1) signal, which promotes interleukin-6 (IL-6) trans-signaling [54], induces vascular wall thickening via activation of the protein kinases [55], impairs mitochondrial function [56], and generates reactive oxygen species (ROS) [57]. A recent study revealed that certain segments of the S-protein can induce the formation of amyloid, a fibrous protein that is insoluble in water. This protein plays a significant role in blood coagulation and fibrinolytic disorders [58]. Anti-spike protein antibodies bind to the S-proteins that emerge on cell surfaces, which triggers autoimmune inflammatory reactions [59-63]. In addition, the injection of LNPs into mice has been reported to cause strong inflammation [64]. All these findings suggest that the COVID-19 mRNA-LNP vaccine poses a risk of thrombosis in individuals with cancer and might explain the excess mortalities after mass vaccination.

Suppression of cancer immunosurveillance 

Some studies have shown that type I interferon (INF) responses, which play an essential role in cancer immunosurveillance, are suppressed after SARS-CoV-2 mRNA-LNP vaccination [65,66]. A large number of exosomes containing microRNA (miRNA)-148a and miRNA-590 are released from cells where large amounts of S-protein were translated, and each miRNA suppresses the ubiquitin-specific peptidase 33 (USP33)-interferon regulatory factor (IRF9) axis in microglia, which internalize these exosomes [67]. In a review, Seneff et al. explained that this suppresses the function of type I IFN and BRCA2, which are critical factors against cancer cells [26]. Programmed death-ligand1 (PD-L1)/programmed cell death 1 (PD-1) expression in the tumor microenvironment suppresses cancer immunosurveillance profoundly [68]. One study showed that S-protein exposure increases surface expression of PD-L1 on a wide range of immune cell types and tumor cells, and PD-1 on T cells, which suppresses the activity of CD4+ and CD8+ T cells against cancer cells [69]. Another study found that non-cancer-specific IgG4 inhibits the antibody effector functions mediated by cancer-specific IgG1, as evidenced by the dramatic acceleration of growth observed in implanted colorectal and breast tumors and skin papillomas caused by carcinogens following local administration of non-cancer-specific IgG4 [70]. According to a meta-analysis in all cancers, pancreatic cancer, and lymphoma, standardized incidence ratios (SIRs) of patients with IgG4-related disease (IgG4-RD) to the general population were 2.57 (95%CI: 1.72, 3.84), 4.07 (1.04, 15.92), and 69.17 (3.91, 1,223.04), respectively [71]. In another study, anti-spike IgG4 levels rose in the serum of SARS-CoV-2 mRNA vaccine recipients after the second dose and increased further after the third dose [72]. A review on IgG4 discussed how long-term exposure to large amounts of specific antigens, such as those found in SARS-CoV-2 mRNA vaccines, may cause uncontrolled growth of cancer cells through a class switch from IgG1 or IgG3 to IgG4 [73]. Another study showed that IL-10 release with non-specific stimulation in fresh whole blood of recipients of the second dose of BNT162b2 or mRNA-1273 increased within two weeks [74]. These findings might explain excess mortality for all cancers, especially excess deaths for pancreatic cancer and breast cancer in our study.

The SARS-CoV-2 vaccine has been shown to cause immunosuppression and lead to the reactivation of latent viruses such as varicella-zoster virus (VZV, human herpesvirus 3; HHV3) or human herpesvirus 8 (HHV8) in some cases [75,76]. HHV8 is considered oncogenic and can cause Kaposi's sarcoma. Oropharyngeal cancer is reported to be caused by the Ebstein-Barr virus (EBV, HHV4) or human papillomavirus (HPV) [77], which also may be reactivated by possible immunosuppression resulting from vaccination. These phenomena could also help explain the excess deaths from lip/oral/pharyngeal cancer in 2022 when mass vaccination with third and later doses was underway.

Cancer development by SARS-CoV-2 mRNA vaccine

In our study, the AMRs of ovarian cancer, leukemia, prostate, lip/oral/pharyngeal, pancreatic, and breast cancers increased significantly beyond the predicted rates, especially in 2022. All of these cancers are known as estrogen and estrogen receptor alpha (ERα)-sensitive cancers [78-83]. Recent research by Solis et al. on the binding ability of S-protein of SARS-CoV-2 against over 9,000 human proteins has shown that S-protein specifically binds to ERα and upregulates the transcriptional activity of ERα. The addition of estradiol (E2) to human breast cancer cells causes proliferation of the cancer cells, whereas the addition of raloxifene, a selective ERα modulator, inhibits proliferation. Breast cancer cells grow when S is added instead of E2, and the addition of raloxifene inhibits their growth. Solis et al. also mentioned that the finding of S-ERα cytosolic colocalization may lead to a potentiation of membrane-bound ERα signaling [84]. Membrane-bound ERα has been implicated in many pathways, including the activation of c-Myc, which promotes the cell cycle and impacts cancer development [85].

ERα-mediated transcription may induce endogenous DNA double-strand breaks (DSBs) in ER-sensitive cancers [86]. Studies have shown that transcriptionally activated ERα induces DSBs by topoisomerase II and the recently known R-loop/G-quadruplex structures formation, significantly increasing the need for BRCA1 for their repair in breast cancer cells [87-89]. One study showed nuclear translocation of mRNA and S protein with the nuclear localization signal [90], and an in silico bioinformatic analysis showed interactions between the S2 subunit of S-protein and BRCA1, BRCA2, and P53 [91], possibly resulting in their sequestration and dysfunction. The possible co-occurrence of high BRCA1 demand to repair DNA damage caused by activated transcription via ERα bound with S-protein along with dysfunction of BRCA1 sequestrated by S-protein raises concerns about increased cancer risk in ERα-sensitive cells in mRNA-LNP SARS-CoV-2 vaccine recipients.

As mentioned above, there is also great concern about the risk of dysfunction in the crucial cancer suppressor genes, brca2 and P53, as well as BRCA1, through mechanisms involving downregulation of IRF9 through interference by specific miRNA in exosomes [26] and the possible sequestration by the S2 subunit of S-protein in the vaccine [91]. Impaired BRCA1 activity is associated with higher risk of breast, uterine, and ovarian cancer in women and prostate cancer in men, as well as moderately higher risk of pancreatic cancer in both men and women [92]. BRCA2-associated cancers include breast and ovarian cancer in women, prostate and breast cancer in men, and acute myeloid leukemia in children [26]. These findings are highly consistent with our results. 

Additional factors that may contribute to the development of cancer are being investigated. Since endogenous ROS causes oxidative DNA damage [93], excessive oxidative stress resulting from the downregulation of ACE2 by S-protein [57] may contribute to cancer development. One study showed that the downregulation of the Mas receptor promotes the metastasis of epithelial ovarian cancer [94]. ACE2 receptor, bound by S-protein after mRNA-LNP vaccination, may directly cause downregulation and subsequent dysfunction of the Mas receptor, possibly leading to an increased risk of metastasis in vaccinated women with ovarian cancer. The observation that injected LNPs accumulate particularly in the ovaries and bone marrow [38] could better explain our findings of excess mortalities from ovarian cancer and leukemia in 2022. According to an analysis of scientific literature about sex hormone receptors in head and neck squamous cell carcinoma (HNSCC), ERα plays various roles in the biopathology of HNSCC, particularly oropharyngeal cancer. These include promoting DNA hypermutation, facilitating HPV integration, and cooperating with epithelial growth factor receptor (EGFR) [82]. This may explain the increased mortality of lip/oral/pharyngeal cancer in our study.

A recent study showed that SARS-CoV-2 RNA could be reverse-transcribed to DNA and integrated into the human cell genome in vitro [95]. Another study reported that transfected mRNA in the human cells exposed to BNT162b2 leads to unsilencing of the endogenous retrotransposon long interspersed element-1 (LINE-1) and reverse transcription of vaccine mRNA sequences to DNA in the nucleus [96]. Accumulation of vaccine mRNA and reverse-transcribed DNA molecules in the cytoplasm could be expected to induce chronic autoinflammation, autoimmunity, DNA damage, and cancer risk in susceptible individuals [97].

The U.S. Food and Drug Administration (FDA) states in its guidance for the production of viral vaccines for infectious disease, "There are several potential mechanisms by which residual DNA could be oncogenic, including the integration and expression of encoded oncogenes or insertional mutagenesis following DNA integration" [98]. The FDA's guidelines are essential for Japan because Japan's special emergency use authorization depended on FDA approval during the COVID-19 pandemic [99]. Recently, some researchers have reported that several lots of Pfizer-BioNTech and Moderna vaccines contain a certain amount of double-stranded DNA fragments from residual plasmid vectors [100,101]. Some of them mentioned that the amount of residual DNA exceeds the regulatory limits for residual DNA set by the FDA. Given these reports and the FDA's regulatory statement, further investigation is required to determine whether the observed excess cancer deaths following mass vaccination were linked to reported residual DNA in the vaccine.

Limitations

This study was conducted using descriptive statistics from official sources and has not been clinically validated. Further analytical statistics study by vaccination status is needed.

## Conclusions

Statistically significant increases in age-adjusted mortality rates of all cancer and some specific types of cancer, namely, ovarian cancer, leukemia, prostate, lip/oral/pharyngeal, pancreatic, and breast cancers, were observed in 2022 after two-thirds of the Japanese population had received the third or later dose of SARS-CoV-2 mRNA-LNP vaccine. These particularly marked increases in mortality rates of these ERα-sensitive cancers may be attributable to several mechanisms of the mRNA-LNP vaccination rather than COVID-19 infection itself or reduced cancer care due to the lockdown. The significance of this possibility warrants further studies. This article was previously posted to the Zenodo repository server on September 18, 2023.
